The article "Combination of Tanshinone IIA and Cisplatin Inhibits Esophageal Cancer by Downregulating NF-κB/COX-2/VEGF Pathway" was retracted in 2021. Reason: concerns about the images.

# Combination of Tanshinone IIA and Cisplatin Inhibits Esophageal Cancer by Downregulating NF-κB/COX-2/VEGF Pathway

**DOI:** 10.3389/fonc.2020.01756

**Published:** 2020-09-10

**Authors:** Xiaozhong Liao, Ying Gao, Jiahui Liu, Lanting Tao, Dongmei Wang, Dan Xie, Suilin Mo

**Affiliations:** ^1^Department of Traditional Chinese Medicine, The First Affiliated Hospital, Sun Yat-sen University, Guangzhou, China; ^2^The State Key Laboratory of Oncology in South China, Sun Yat-sen University Cancer Center, Collaborative Innovation Center for Cancer Medicine, Guangzhou, China; ^3^Department of Oncology, The First Affiliated Hospital of Guangzhou University of Chinese Medicine, Guangzhou, China; ^4^School of Pharmaceutical Sciences, Sun Yat-sen University, Guangzhou, China

**Keywords:** Tan IIA, DDP, synergistic effect, ESCC, NF-κB/COX-2/VEGF pathway

## Abstract

Cisplatin (DDP) represents one of the common drugs used for esophageal squamous cell carcinoma (ESCC), but side effects associated with DDP and drug resistance lead to the failure of treatment. This study aimed to understand whether tanshinone IIA (tan IIA) and DDP could generate a synergistic antitumor effect on ESCC cells. Tan IIA and DDP are demonstrated to restrain ESCC cell proliferation in a time- and dose-dependent mode. Tan IIA and DDP at a ratio of 2:1 present a synergistic effect on ESCC cells. The combination suppresses cell migration and invasion abilities, arrests the cell cycle, and causes apoptosis in HK and K180 cells. Molecular docking indicates that tan IIA and DDP could be docked into active sites with the tested proteins. In all treated groups, the expression levels of E-cadherin, β-catenin, Bax, cleaved caspase-9, P21, P27, and c-Fos were upregulated, and the expression levels of fibronectin, vimentin, Bcl-2, cyclin D1, p-Akt, p-ERK, p-JNK, P38, COX-2, VEGF, IL-6, NF-κB, and c-Jun proteins were downregulated. Among these, the combination induced the most significant difference. Our results suggest that tan IIA could be a novel treatment for combination therapy for ESCC.

## Introduction

Esophageal cancer (EC) represents the sixth most deadly cancer (1). Esophageal squamous cell carcinoma (ESCC) accounts for the majority of EC and is the fourth leading cause of cancer death in China (2). Currently, the clinical approach for ESCC is surgical treatment combined with chemoradiotherapy. Chemotherapy is a critical treatment for ESCC and has been shown to provide specific therapeutic effects (3, 4). Furthermore, cisplatin (DDP)-based chemotherapy is the standard first-line treatment for ESCC (5). Unfortunately, the 5-year overall survival rate remains very poor, and side effects and acquired drug resistance remain major clinical obstacles that must be overcome in order to achieve successful treatment (6–8).

DDP has the molecular formula Cl_2_H_6_N_2_Pt and a molecular mass of 300 g/mol. The compound ID (CID) of DDP in PubChem Compound is 441203 (Figure 1B). It has been extensively utilized to cure different types of neoplasms, including head and neck (9, 10), lung (11, 12), ovarian (13, 14), breast (15, 16), brain (17, 18), kidney (19, 20), and esophagus cancers (21–23). In general, DDP and other platinum-based compounds are considered to be cytotoxic drugs, which can induce apoptosis of cancer cells (24). Numerous molecular anticancer mechanisms have been described, including the induction of p53 signaling and cell cycle arrest (25, 26), downregulation of proto-oncogenes and anti-apoptotic proteins, and activation of both intrinsic and extrinsic apoptosis (27, 28). However, DDP has also been associated with substantial side effects, including hepatotoxic, nephrotoxic, cardiotoxic, neurotoxic, and/or hematotoxic damage. In addition, acquired resistance often leads to failure of DDP chemotherapy. Currently, combination therapies of DDP with other drugs are commonly used in clinical treatment. Several studies have indicated that the combination of DDP with other drugs represents the best therapeutic approach for overcoming drug resistance and reducing undesirable side effects (29). A combination strategy can be a possible new choice for clinical treatment.

**FIGURE 1:** 2D structure of Tan IIA **(A)** and DDP **(B)** (obtained from PubChem compound http://pubchem.ncbi.nlm.nih.gov/).

Tanshinone IIA (tan IIA) has the molecular formula C_19_H_18_O_3_ and a molecular mass of 294.344420 g/mol (Figure 1A). Tan IIA represents one of the primary fat-soluble compositions isolated from Salvia miltiorrhiza, referred to as “dan-shen” in traditional Chinese medicine (30). The CID of tan IIA in PubChem Compound is 164676. The anticancer effects of tan IIA in a wide range of cancer cells have been studied *in vitro*, including lung (31), liver (32), stomach (33), and pancreatic cancer cells (34). Our previous studies demonstrate that tan IIA functioned to inhibit the growth of NSCLC A549 cells by decreasing VEGF/VEGFR2 expression (35). It has been demonstrated that the combination of tan IIA and adriamycin (ADM) not only exhibits a synergistic effect on HepG2, but also improves the cytotoxicity of ADM with less cardiotoxicity (32). In addition, it has been demonstrated that tan IIA could function to protect cardiomyocytes from ADM-induced apoptosis, in part, through Akt-signaling pathways (36). These studies prompted the idea that tan IIA could improve the cytotoxicity of DDP and function as an effective adjunctive reagent in ESCC treatment. However, the effect of tan IIA in combination with DDP on ESCC cells remains unclear.

Therefore, we aimed to explore whether tan IIA and DDP could induce a synergistic antitumor effect in ESCC cells and clarify the potential molecular mechanisms based on the drug–protein interaction analysis platform built up in our previous studies (37, 38).

## Results

### Tan IIA and DDP Synergistically Inhibit the Growth of the ESCC Cells

We first observed the effect of either tan IIA or DDP on the proliferation of ESCC cells, and we found that both tan IIA and DDP could individually inhibit ESCC cell proliferation in a time- and concentration-dependent manner. The 48 h 50% inhibitory concentration (IC_50_) values of tan IIA for HK (Figure 2A), K180 (Figure 2C), EC109 (Figure 2E), and K70 (Figure 2G) cell lines were 5.81, 6.00, 3.42, and 6.31 μM, respectively, and the IC_50_ values of DDP were 2.41, 1.98, 2.37, and 2.81 μM, respectively.

**FIGURE 2:** The proliferative inhibition effect of Tan IIA, DDP, and the combination treatment on ESCC cells. Drug concentration-Cell viability curves were generated as the viable cell percentage based on the cell viability assay **(A,C,E,G)**. Synergistic effects between Tan IIA and DDP were exhibited as Fa-CI plots **(B,D,F,H)**. Data are from three repeated experiments with quadruplicate wells, (mean ± SD).

Based on the IC_50_ values, we set up the combination treatment at ratio of 2:1 (tan IIA:DDP) for 48 h treatment. In comparison with a single drug, the combination a generated greater inhibitory effect on cancer cell proliferation. The synergism of the combination was observed in HK (Figure 2B), K180 (Figure 2D), and EC109 (Figure 2F) cells, no matter what the fraction affected value was (Fa range: 0–1, where Fa = 0 represents 100% viability and Fa = 1 represents 0% viability). The combination of tan IIA and DDP exhibited a synergistic inhibitory effect on K70 (Figure 2H) cells when the Fa value was ≤0.877. The summary of combination index (CI) and the concentrations of the drugs used in combination at 50% Fa are depicted in Table 1.

**TABLE 1:** Summary of CI value and the concentration of separate drugs in combination at 50% Fa.

Drug combination	Fa = 0.5			
	
	HK	K80	EC109	K70
**DDP + Tan IIA**				
CI	0.58033	0.65037	0.66513	0.61702
DDP (μm)	0.82640	0.82134	0.93801	0.95273
Tan IIA (μm)	1.65280	1.64268	1.87602	1.90546

### Tan IIA and DDP Inhibit Migration and Invasion of the ESCC Cells

We next explored the effect of either individual or combined tan IIA and DDP treatment on cancer cell migration and invasion. We utilized wound healing and transwell assays to evaluate the migration and invasion abilities of HK and K180 cells. Results show that both the migration distance (Figures 3A,B) and invasive cell numbers (Figures 3C,D) were significantly decreased following a 24-h drug treatment. Furthermore, the tan IIA and DDP combination treatment exhibited the strongest inhibition on cell migration and invasion (Figures 3E–H). We next used molecular docking to study the potential interactions between the drugs and epithelial–mesenchymal transition (EMT)-related proteins, such as E-cadherin, β-catenin, fibronectin, and vimentin. Results show that both tan IIA and DDP could be docked into the active site of fibronectin in its binding pocket (Figures 3I–M). Tan IIA was shown to be able to form H-bonds with TRP 146 and CYS 148 and π-π interactions with LEU 134, CYS 148, and PRO 150 in the site within fibronectin in 10 random poses (Figures 3J,K), and DDP was found to form H-bonds with CYS 148 (Figures 3L,M). In addition, we carried out western blotting analyses to study changes in EMT-related proteins. Results indicate that, following a single drug treatment of HK (Figures 3N,P,Q) and K180 (Figures 3O,R,S) cells, the expression levels of the epithelial markers E-cadherin and β-catenin were significantly increased, and the expression levels of the mesenchymal markers fibronectin and vimentin were decreased. Notably, the drug combination treatment exhibited the most significant effect in comparison to the individual drug treatments. These findings demonstrate that the tan IIA and DDP combination treatment could significantly affect the expression levels of EMT-related proteins, but the specific mechanism of the drug–protein interaction is still unclear.

**FIGURE 3:** Tan IIA and DDP suppressed migration and invasion ability of ESCC cells. Representative images of wound healing and transwell assay in HK **(A,C)** and K180 **(B,D)** cells following 24 h treatment with 6 μM Tan IIA, 3 μM DDP alone and 1 μM DDP and 2 μM Tan IIA in combination. Histograms depict the average migrated distance and the number of invasive cells in HK **(E,F)** and K180 **(G,H)** cells, respectively. The 3D crystal structure of human Fibronectin with an endogenous ligand (PDB-ID: 2cg6) **(I)**. Ten random poses of Tan IIA docked into the active site of 2cg6 **(J)**. The binding modes of Tan IIA in Fibronectin: at least five residue involved in the interactions in ten random poses, TRP 146, CYS 148 (H-bonds) and LEU 134, CYS 148, PRO 150 (π-π interaction) **(K)**. Ten random poses of DDP docked into the same active site of 2cg6 **(L)**. The binding modes of DDP in Fibronectin: at least one residue involved in the interactions in ten random poses, CYS 148 (H-bonds) **(M)**. Protein expression levels of E-cadherin, β-catenin, Fibronectin, Vimentin and GAPDH of HK and K180 cells following a 48 h treatment with 6 μM Tan IIA, 3 μM DDP alone and 1 μM DDP and 2 μM Tan IIA in combination **(N,O)**. Histograms depict the relative gray value of the related proteins measured using Image J **(P–S)**. All data are shown as the mean ± SD of three independent experiments. **P < 0.01, ***P < 0.001, or ****P < 0.0001 versus the control group (magnification, ×100, Scale bars, 100 μm).

### Tan IIA and DDP Arrest Cell Cycle of the ESCC Cells

Following verification of the antiproliferation effect of tan IIA and DDP, we utilized flow cytometry to analyze the cell cycle of the treated ESCC cells. As shown in Figures 4A–D, compared with control groups, all of the treatment groups showed increased S and G2 phase cell populations, and the combination treatment was found to be more significant than the individual treatments. Then, we applied molecular docking to investigate the interactions between the drugs and P21 (Figure 4E). The results show that both tan IIA (Figure 4F) and DDP (Figure 4H) could be docked into the active site of P21 (Figure 4E) in the binding pocket. Tan IIA was shown to be able to form H-bonds with ASP 156, ALA 208, ARG 210, and π-π interactions with ALA 208 and ARG 210 in the site within P21 (Figure 4G), and DDP was found to form H-bonds with ASP 156 and ARG 210 (Figure 4I). In addition, western blotting analyses demonstrated that, following the single drug treatments in HK (Figures 4J,L) and K180 (Figures 4K,M) cells, the expression levels of P21 and P27 increased, and the expression levels of cyclin D1 decreased. Again, the combination treatment demonstrated the most significant effect. However, the specific mechanism of the drug–protein interaction is still unclear. These findings suggest that combination treatment of tan IIA and DDP could affect cell cycle arrest in the S and G2 phases.

**FIGURE 4:** Effect of Tan IIA and DDP alone and in combination on cell cycle arrest. The percentage of cells in G1, S or G2/M phase in HK **(A)** or K180 cells **(C)** treated with 6 μM Tan IIA, 3 μM DDP alone and 1 μM DDP and 2 μM Tan IIA in combination for 24 h. Data represent the cell population of cell cycle arrest of HK **(B)** and K180 **(D)** cells. The 3D crystal structure of human P21 with an endogenous ligand (PDB-ID: 2zvw) **(E)**. Ten random poses of Tan IIA docked into the active site of 2zvw **(F)**. The binding modes of Tan IIA in P21: at least five residue involved in the interactions in ten random poses, ASP 156, ALA 208, ARG 210 (H-bonds) and ALA 208, ARG 210 (π-π interaction) **(G)**. Ten random poses of DDP docked into the same active site of 2zvw **(H)**. The binding modes of DDP in P21: at least two residue involved in the interactions in ten random poses, ASP 156, ARG 210 (H-bonds) **(I)**. Protein expression levels of Cyclin D1, p21, p27, and GAPDH of HK **(J)** and K180 **(K)** cells following 24 h treatment with 6 μM Tan IIA, 3 μM DDP alone and 1 μM DDP and 2 μM Tan IIA in combination. Histograms represent the relative gray value of the related proteins measured by Image J **(L,M)**. All data are depicted as the mean ± SD of three independent experiments. *P < 0.05, **P < 0.01, ***P < 0.001, or ****P < 0.0001 versus the control group.

### Tan IIA and DDP Induce Apoptosis of the ESCC Cells

As depicted in Figure 5, all treatment groups were found to increase the proportion of early (right lower quadrant) and late apoptosis (right upper quadrant) in HK (Figures 5A,B) and K180 (Figures 5C,D) cells. In addition, combination treatment was found to more potently induce apoptosis in comparison with the single treatments in HK and K180 cells. In Figures 5E–I, we applied molecular docking to seek the interactions between the drugs and Bcl-2 (Figure 5E). The results indicate that tan IIA (Figure 5F) and DDP (Figure 5H) could be docked with Bcl-2. Tan IIA formed H-bonds with TYR 199 and π-π interactions with TYR 105, LEU 134, and ALA 146 in the site within Bcl-2 (Figure 5G), and DDP formed H-bonds with GLY 142 and TYR 199 and π-π interactions with TYR 105, LEU 134, and ALA 146 (Figure 5I). We also carried out western blotting analyses to examine the levels of apoptosis-related proteins. The relative density values demonstrated that, following the single drug treatment in HK (Figures 5J,L) and K180 (Figures 5K,M) cells, the expression levels of cleaved caspase-9 and Bax increased, and the expression level of Bcl-2 decreased. Again, the combination treatment showed the most significant effect. However, the specific mechanism of the drug–protein interaction is still unclear. These findings suggest that the combination treatment of tan IIA and DDP could induce ESCC cell apoptosis.

**FIGURE 5:** Effect of Tan IIA, DDP alone and in combination on apoptosis. Representative profiles showing apoptosis in HK **(A)** or K180 cells **(C)** treated with 6 μM Tan IIA, 3 μM DDP alone and 1 μM DDP and 2 μM Tan IIA in combination for 48 h. Data represent the cell population of cell cycle arrest of HK **(B)** and K180 **(D)** cells. The 3D crystal structure of human Bcl-2 with an endogenous ligand (PDB-ID: 4lvt) **(E)**. Ten random poses of Tan IIA docked into the active site of 4lvt **(F)**. The binding modes of Tan IIA in Bcl-2: at least four residues involved in the interactions in ten random poses, TYR 199 (H-bonds) and TYR 105, LEU 134, ALA 146 (π-π interaction) **(G)**. Ten random poses of DDP docked into the same active site of 4lvt **(H)**. The binding modes of DDP in Bcl-2: at least five residues involved in the interactions in ten random poses, ASN 142, TYR 199 (H-bonds) and TYR 105, LEU 134, ALA 146 (π-π interaction) **(I)**. Protein expression levels of Cleaved casp9, Bcl-2, Bax, and GAPDH of HK **(J)** and K180 **(K)** cells following 48 h treatment with 6 μM Tan IIA, 3 μM DDP alone and 1 μM DDP and 2 μM Tan IIA in combination. Histograms depict the relative gray value of the related proteins measured using Image J **(L,M)**. All data are shown as the mean ± SD of three independent experiments. **P < 0.01 or ****P < 0.0001 versus the control group.

### Tan IIA and DDP Inhibit ESCC Xenograft Tumor Growth

We next explored the influence of tan IIA and DDP on ESCC *in vivo* (Figure 6A). As shown in Figure 6B, tan IIA has no significant influence on the body weight of mice compared with the control group and can weaken the effect of DDP on the body weight loss of mice. We also performed H&E staining after embedding sections of the organs, and found that the drugs had no obvious toxic and side effects on the heart, lung, liver, kidney, and brain tissues (Supplementary Figure S1). In the control group, xenograft tumors grew faster than the treatment groups (Figure 6E), and the tumor volume and weight in the normal saline group was observed to be significantly larger than those in the treatment groups (Figures 6C,D). In comparison with the single-drug treatment, the combination group was found to inhibit tumor growth more significantly. Taken together, this suggests that tan IIA could strengthen the antitumor effect of DDP *in vivo*.

**FIGURE 6:** Tan IIA, DDP alone and in combination suppress the growth of K180 cells *in vivo*. Timeline of K180 cells inoculation and drug treatment **(A)**. Time courses of animal weight **(B)**. Tumor volume of all groups was measured every 4 days, beginning the first day after injection until the study end point. Data are shown as growth curves **(C)**. Tumor mass of all groups was measured and compared, ***P < 0.001 versus the control group **(D)**. Tumors derived from K180 cells in six male nude mice are presented **(E)**.

### Binding Patterns of Tan IIA and DDP With the Tested Proteins

The AKT and ERK pathways have been demonstrated to play critical roles in cancer proliferation and metastasis. COX-2 has been shown to be a key molecular regulator of cancer progression and metastasis and a crucial target in cancer therapy. A recent study found that tan IIA could downregulate COX-2 expression and inactivate the NF-κB pathway in SH-SY5Y cells (39). Therefore, we used molecular docking for further research. The 3-D crystal structures of AKT, JNK, P38, and VEGF are depicted in Figures 7A,F,K,P. All of the structures are shown with an endogenous ligand. In Table 2, the root mean square deviation (RMSD) values of fibronectin, P21, Bcl-2, AKT, JNK, P38, and VEGF were 1.591, 0.977, 2.001, 0.939, 1.156, 0.646, and 1.786 Å, respectively. This indicates that the CDOCKER module had a higher veracity compared to LibDock. Therefore, the CDOCKER module was chosen for study.

**FIGURE 7:** Interactions between the drugs and the NF-κB/COX-2/VEGF axis signaling pathway. 3D crystal structure of human AKT with an endogenous ligand (PDB-ID: 3d0e) **(A)**, Ten random poses of Tan IIA docked into the active site of 3d0e **(B)**. The binding modes of Tan IIA in AKT, at least three residues involved in the interactions in ten random poses, LYS 160 (H-bonds) and VAL 166, ALA 179 (π-π interaction) **(C)**. Ten random poses of DDP docked into the same active site of 3d0e **(D)**. The binding modes of DDP in AKT, at least five residues involved in the interactions in ten random poses, GLU 236, GLU 279, ASP 293, and ASP 964 (H-bonds), and LEU 158, VAL 166 (π-π interaction) **(E)**. 3D crystal structure of human JNK with an endogenous ligand (PDB-ID: 4y46) **(F)** Ten random poses of Tan IIA docked into the active site of 4y46 **(G)**. The binding modes of Tan IIA in JNK, at least eight residues involved in the interactions in ten random poses, MET 149 (H-bonds) and ILE 70, VAL 78, ALA 91, MET 146, MET 149, VAL 196, LEU 206 (π-π interaction) **(H)**. Ten random poses of DDP docked into the same active site of 4y46 **(I)**. The binding modes of DDP in JNK, at least seven residues involved in the interactions in ten random poses, MET 146, GLU 147, MET 149, ASP 150, ASN 152, GLN155 (H-bonds), and VAL 78 (π-π interaction) **(J)**. The 3D crystal structure of human P38 with an endogenous ligand (PDB-ID: 2YIX) **(K)** Ten random poses of Tan IIA docked into the active site of 2YIX **(L)**. The binding modes of Tan IIA in P38, at least eight residues involved in the interactions in ten random poses, GLU 71, LEU108, MET 109, GLY 110, LEU 167, ASP 168 (H-bonds) and VAL 30, TYR 35, LEU 108 (π-π interaction) **(M)**. Ten random poses of DDP docked into the same active site of 2YIX **(N)**. The binding modes of DDP in P38, at least five residues involved in the interactions in ten random poses, GLU 71, MET 109, GLY 110, LEU 167, ASP 168 (H-bonds), and VAL 30, TYR 35, LEU 108 (π-π interaction) **(O)**. 3D crystal structure of human VEGF with an endogenous ligand (PDB-ID: 5hhc) **(P)**, Ten random poses of Tan IIA docked into the active site of 5hhc **(Q)**. The binding modes of Tan IIA in VEGF, at least four residues involved in the interactions in ten random poses, GLY 52, GLU 60, CYS 61 (H-bonds) and CYS 53 (π-π interaction) **(R)**. Ten random poses of DDP docked into the same active site of 5hhc **(S)**. The binding modes of DDP in VEGF, at least three residues involved in the interactions in ten random poses, GLY 51, GLY 52 and CYS 61 (H-bonds) **(T)**.

**TABLE 2:** The validation of molecular docking algorithm (RMSD).

Protein	CDOCKER RMSD (Å)	LibDock RMSD (Å)
(Fibronectin) 2CG6	1.591	*
(P21) 2ZVW	0.977	*
(Bcl-2) 4IEH	2.001	6.850
(AKT) 3D0E	0.939	2.608
(JNK) 4Y46	1.156	4.695
(P38) 2YIX	0.646	1.986
(VEGF) 5HHC	1.786	*

*In LibDock module, both Tan IIA and Cisplatin cannot dock with the targeted protein.

In Figure 7, two drugs can be docked with AKT (Figures 7B–E), JNK (Figures 7G–J), P38 (Figures 7L–O), and VEGF (Figures 7Q–T). These suggest that tan IIA and DDP could interact with the tested proteins in different ways, thereby influencing the NF-κB/COX-2/VEGF signaling pathway, which could be the underlying molecular mechanism responsible for the synergy of tan IIA and DDP. However, the specific mechanism of the drug–protein interaction is still unclear.

### Tan IIA and DDP Downregulate the NF-κB/COX-2/VEGF Signaling Pathway in the ESCC Cells

In order to explore the relevant signaling pathway, we used western blotting to quantify the expression levels of p-Akt, Akt, p-ERK, ERK, p-JNK, JNK, P38, COX-2, VEGF, IL-6, NF-κB, c-Jun, and c-Fos in K180 cells treated with tan IIA and DDP alone and also in combination. As shown in Figures 8A–F, the expression levels of p-Akt, p-ERK, p-JNK, P38, COX-2, VEGF, IL-6, NF-κB, and c-Jun were downregulated in all of the treatment groups. However, the expression levels of c-Fos protein were observed to be upregulated, and the total levels of Akt, ERK, JNK, and GAPDH levels were unchanged. The combination exhibited the most significant effect in comparison with the single drug.

**FIGURE 8:** Suppressive effect of Tan IIA, DDP, and the combination on NF-κB/COX-2/VEGF axis signaling pathway in K180 cells. Protein expression levels of p-Akt, Akt, p-ERK, ERK, p-JNK, JNK, p38, COX-2, VEGF, IL-6, NF-κB, c-Jun, c-fos and GAPDH in K180 cells treated with 6 μM Tan IIA, 3 μM DDP alone and 1 μM DDP and 2 μM Tan IIA in combination for 48 h **(A,B)**. Histograms depict the relative gray value of the related proteins measured using Image J **(C–F)**. All data are shown as the mean ± SD of three independent experiments. *P < 0.05, **P < 0.01, ***P < 0.001, or ****P < 0.0001 versus the control group.

## Discussion

The National Comprehensive Cancer Network guidelines recommend the use of combinational drugs for treatment of ESCC, including DDP combined with ADM and 5-fluorouracil (5-Fu). However, the most critical difficulties associated with ESCC treatment are the side effects and intrinsic resistance (40). Therefore, profound discoveries and a greater understanding of its mechanism of action could lead to the generation of novel therapies to overcome DDP chemoresistance and ultimately improve the survival of ESCC patients.

Small molecules extracted from Chinese herbal medicine have been reported to reverse the chemoresistance of cancers (41–44). Increasing reports demonstrate that tan IIA possesses therapeutic potential for numerous diseases with few side effects (30, 32–34, 36, 38). Among the numerous biological activities of tan IIA, greater attention has been focused on increasing the sensitivity of tumor cells to chemotherapeutic drugs (45, 46). Our previous studies demonstrate that the combination of tan IIA with ADM functions to inhibit the malignant biological behaviors of NSCLC cells in a synergistic way and was able to enhance the antitumor effect of ADM (38). These findings suggest that tan IIA could be developed as a novel agent for postoperative adjuvant therapy via combination with other antitumor agents.

Although tan IIA has been utilized as an antitumor agent for different cancers, the effect of tan IIA in combination with DDP on ESCC cells remains largely unclear. In this study, we find that tan IIA and DDP exert inhibitory effects on the growth of ESCC cells in a concentration- and time-dependent mode (Figure 2). However, the effect of tan IIA was found to be weaker than that of DDP. Further experiments demonstrate that the combination can function to suppress cell migration and invasion, arrest the cell cycle, and induce apoptosis in HK and K180 cells. Furthermore, we certify the mechanisms of tan IIA and DDP in HK and K180 cells by downregulating the NF-κB/COX-2/VEGF signaling pathway.

It has been demonstrated that tan IIA could suppress the migration and invasion of breast and bladder cancer (47, 48), which is consistent with our findings that tan IIA and DDP restrained the migration and invasion of ESCC cells, and the combined treatment exerted a greater inhibitory effect (Figures 3A–H). Moreover, tan IIA upregulated the epithelial markers E-cadherin and β-catenin and downregulated mesenchymal markers, such as fibronectin and vimentin in a time- and dose-dependent manner (47, 48). We also found that tan IIA could influence the expression of EMT-related proteins, and the combination of these two drugs exerted a greater effect (Figures 3N–S). This indicates that the combination could decrease ESCC cell invasiveness through inhibition of EMT. However, the specific mechanism of the drug–protein interaction is still unclear, and more molecular biology experiments are needed to further study the specific interaction mechanism between drugs and proteins in the future.

Our previous research demonstrates that, in A549 cells, S- and G2-phase cells were overtly aggrandized after tan IIA treatment (38). Consistently, we also observed that tan IIA and DDP could arrest ESCC cells at the S and G2 phases. Combined treatment was found to have more significant results (Figures 4A–D). Western blotting analyses demonstrate that the combination affects the expression of cell cycle–related proteins (Figures 4J–M). However, the effect of tan IIA on the cell cycle distribution is still controversial. Ma’s study found that, in the NSCLC cell line H1299, the proportion in the G1 phase was increased following treatment with tan IIA (49). This indicates that low-concentration tan IIA might arrest the cell cycle at the G1 phase, whereas high-concentration tan IIA might lead to S-phase cell cycle blockage, which remains to be further explored. In addition, the specific mechanism of action between drugs and related proteins still needs further verification by molecular biology experiments.

A recent study certified that tan IIA can induce apoptosis of NSCLC cells in a concentration- and time-dependent manner (50). Consistently, our results found that tan IIA and DDP were able to individually induce apoptosis in HK and K180 cells with the combination inducing a significantly higher apoptosis of cancer cells (Figures 5A–D). We preliminarily find that apoptosis may be related to cleaved caspase-9, Bcl-2, and Bax, but the specific mechanism of action between drugs and related proteins has not been clarified yet. A large number of molecular biological experiments are still needed for research.

A xenograft model in mice suggests that tan IIA could function to effectively increase the antitumor effect of DDP *in vivo* (Figure 6). H&E staining indicated that the drugs had no obvious toxic and side effects on the heart, lung, liver, kidney, and brain tissues (Supplementary Figure S1), which is contrary to other relevant research that DDP (10 mg/kg) could induce tubular dilatation, cast formation, and vacuolization in the kidneys (51). This may be due to the fact that we used a lower concentration of DDP (3 mg/kg). However, more animal studies are needed for research.

COX-2, a COX isoform, plays critical roles in carcinogenesis. Extensive evidence accumulated over the past several decades suggests that COX-2 expression is enhanced in numerous premalignant tissues and malignant tumors, including Barrett’s esophagus and esophageal cancer (52, 53). Further studies demonstrate that COX-2 overexpression is associated with angiogenesis as well as tumor invasion and metastasis (54). COX-2 has also been found to be able to modulate P-glycoprotein (MDR-1), which contributes to drug resistance (55). COX-2-derived PGs have been shown to play a critical role in the regulation of esophageal tumor cell proliferation and apoptosis (56). Therefore, COX-2 inhibition could be useful for the treatment of esophageal cancer. Tan IIA could downregulate COX-2 expression and inactivate the NF-κB pathway in SH-SY5Y cells (39).

Our study also utilizes molecular docking, which is applied in our other studies (35, 38, 57–59) to detect interactions present between drugs and proteins involved in the NF-κB/COX-2/VEGF signaling pathway. We find that tan IIA and DDP could be docked with the tested proteins, including AKT, JNK, P38, and VEGF. Different binding modes suggest that tan IIA and DDP could possibly affect protein in different ways. However, the specific mechanism of action between drugs and related proteins still needs further verification by molecular biology experiments. Western blotting analyses show that tan IIA and DDP could downregulate the NF-κB/COX-2/VEGF signaling pathway in HK and K180 cells. Therefore, there is a great possibility that tan IIA and DDP could function as anti-ESSC therapies, and the different manners of interaction with the tested proteins inside the NF-κB/COX-2/VEGF signaling pathway might be the underlying molecular mechanisms although further studies are still required to determine the possible mechanisms behind the combination treatment of tan IIA and DDP.

## Materials and Methods

### Materials and Cell Culture

HK, K180, Eca109, and K70 were kindly provided by the State Key Laboratory of Oncology in South China and were grown at 37°C in 5% CO_2_ in a humidified incubator in Dulbecco’s modified eagle’s medium (DMEM) (Invitrogen Corp., Carlsbad, CA, United States) containing 10% fetal bovine serum (Invitrogen Corp., Carlsbad, CA, United States), 100 U/mL penicillin, and 100 U/mL streptomycin (Gino, Hangzhou, Zhejiang, China). Tan IIA and DDP were purchased from Sigma (St. Louis, MO, United States). Tan IIA was dissolved in DMSO (1 mM), and DDP was dissolved in physiological saline (10 mM) and then both of them were stored at −20°C for future use.

### Cell Viability Assay

Drug sensitivity analysis was performed using the cell counting kit-8 (CCK-8) (Dojindo Laboratories, 119 Kumamoto, Japan) according to the manufacturer’s instructions. After incubating cells for 24, 48, or 72 h in 96-well plates at 8000 cells/well with four replicates, different drugs were added (controls received a similar volume of DMEM). Cells were then cultured with 100 μl of fresh medium supplemented with 10 μl of CCK-8 solution, and the plates were further incubated for 1.5 h at 37°C. The optical densities were read on a microplate reader (Thermo Scientific, Rockford, IL, United States) at a wavelength of 450 nm. Here is the formula used to calculated the proliferative inhibition rate: Proliferative inhibition rate = (1- experimental group/control group) × 100%. The 50% inhibitory concentrations (IC_50_) were determined using non-linear regression analysis using SPSS 20.0 software.

### Synergy Determination

The CI and isobologram plot were calculated according to the Chou–Talalay method. Further, the data received from the cell viability assay were transferred into Fa (range from 0 to 1; where Fa = 0 represents 100% viability and Fa = 1 represents 0% viability) and analyzed by the CompuSyn^TM^ program (Biosoft, Ferguson, MO, United States). CI values of <1.0 indicate synergism, and values of >1.0 the opposite.

### Wound Healing Assay

Cells were seeded in complete media into six-well plates (1 × 10^6^ per well). After 24 h, a scratch wound was made using a pipette tip, and the cells were then rinsed three times with PBS. Further cells were cultured with a serum-free medium containing various different groups of drugs for 24 h. After 0 and 24 h, photos (magnification × 10) were acquired at the scratched point. The moving distance of cells was then calculated by Adobe Photoshop CS6 software.

### Transwell Assay

For this assay, 3 × 10^4^ cells were trypsinized and resuspended in serum-free medium containing different drugs and placed in the upper chamber of the transwell insert (8 μm pore, 6.5 mm polycarbonate, Corning, NY, United States) that was covered with a layer of Matrigel Basement Membrane Matrix (BD Biosciences, Bedford, MA, United States) in advance. After 24 h of incubation, the cells were fixed with 4% paraformaldehyde at room temperature for half an hour and dyed with 0.5% crystal violet. The cells on the upper surface of the filter were cleaned with a cotton swab. Finally, the number of dyed cells was calculated using the microscope (magnification × 100). For each transwell filter, a sum of 5 fields was calculated.

### Flow Cytometric Cell Cycle Analysis

The cell cycle was detected by the Cell Cycle Detection Kit obtained from 4A Biotech Co., Ltd., and 1.0 × 10^6^ cells were plated into 6-well plates and treated with full medium containing different drugs for 24 h. Next, cells were harvested, washed with PBS, and fixed in cold 70% ethanol at 4°C overnight. Afterward, cells were washed with PBS, incubated with RNase A at 37°C for half an hour, and then incubated with 400 μl propidium iodide (PI) for 30 min. All cells (at least 50,000 per test) were detected by ACEA NovoCyte flow cytometer equipped with Novoexpress (Becton Dickinson, San Jose, CA, USA) was applied to detect the cell cycle.

### Apoptosis Assay

The annexin V-FITC Apoptosis Detection Kit (4A Biotech Co., Ltd.) was used to detect cell apoptosis. For it, 1.0 × 10^5^ cells were plated into 6-well plates and treated with various drugs for 48 h. Cells in different groups were then collected, cleaned with cold PBS, and then stained with annexin V-FITC and PI for 30 min. After staining, the apoptosis rates were detected immediately using an ACEA NovoCyte flow cytometer equipped with Novoexpress (Becton Dickinson, San Jose, CA, USA) was applied to detect cell *apoptosis*.

### Mice Xenograft Model

Tumor cells in log-phase growth were resuspended in NS, and 10^6^ cells were injected subcutaneously into the right dorsal flank. The tumor volume was defined as follows: V = W^2^L/2, in which W is the shortest diameter and L is the longest diameter. When it reached 300 mm^3^, the mouse began to receive an intraperitoneal injection of equal volume of tan IIA (15 mg/kg), DDP (3 mg/kg), tan IIA (7.5 mg/kg) and DDP (1.5 mg/kg), or normal saline twice a week. All mice were sacrificed, and tumors were harvested at the end point. The animal studies were examined and approved by the SYSUCC Institutional Animal Care and Usage Committee. All procedures were conducted under the Guidelines for the Care and Use of Laboratory Animals (NIH publications Nos. 80-23, revised 1996).

### Molecular Docking

The molecular docking algorithm was carried out in this research with Discovery Studio (DS) 2.5 to have a better understanding of the potential interactions between the tested drugs and the selected proteins. The two-dimensional structures of tan IIA and DDP were from the database of Pubchem^1^, and the PubChem CIDs are, respectively, 164676 and 441203. The 3-D structures of fibronectin (PDB-ID: 2CG6), P21 (PDB-ID: 2ZVW), BCl-2 (PDB-ID: 4LVT), AKT (PDB-ID: 3D0E), JNK (PDB-ID: 4Y46), P38 (PDB-ID: 2YIX), and VEGF (PDB-ID: 5HHC) were acquired from the database of the Protein Data Bank (PDB)^2^. DS 2.5 was used to conduct the virtual docking procedures. First, the water molecules of the tested proteins were removed and refined with CHARMM on the targeted proteins and the ligands. Then, the possible active sites of the tested proteins based on endogenous ligands were automatically discovered with the algorithm. After the drugs and selected ligands were docked into the binding pocket of the tested proteins, the docking modes of the drugs and the tested proteins were determined. The calculation of RMSD was carried out for the verification of the selection of the two modules (CDOCKER and LibDock) in DS 2.5 before performing the procedure.

### Western Blot Analysis

Western blot analysis was done according to the standard protocol. The following primary antibodies were used: E-cadherin, 1:1000; β-catenin, 1:1000; fibronectin, 1:1000; vimentin, 1:1000; cyclin D, 1:1000; P27, 1:1000; P21, 1:1000; cleaved caspase 9, 1:1000; Bcl-2, 1:1000; Bax, 1:1000; p-Akt, 1:1000; Akt, 1:1000; p-ERK, 1:1000; ERK, 1:1000; p-JNK, 1:1000; JNK, 1:1000; P38, 1:1000; COX-2, 1:1000; VEGF, 1:1000; IL-6, 1:1000; NF-κB, 1:500; c-Jun, 1:500; c-Fos, 1:500 and GAPDH, 1:8000.

### Statistical Analysis

Data are presented as mean ± SD, (X ± SD) and assessed by the two-tailed Student’s *t*-test. A *P*-value less than 0.05 was considered statically significant.

## Data Availability Statement

The raw data supporting the conclusion of this article will be made available by the authors, without undue reservation.

## Ethics Statement

The animal study was reviewed and approved by the SYSUCC Institutional Animal Care and Usage Committee.

## Author Contributions

SM and DX designed and guided the study. XL, YG, JL, and LT performed the *in vitro* and *in vivo* experiments. XL and YG wrote the manuscript. DW performed the molecular docking. SM and DX revised the manuscript. All authors read and approved the final manuscript.

## Conflict of Interest

The authors declare that the research was conducted in the absence of any commercial or financial relationships that could be construed as a potential conflict of interest.

## Footnotes

1 http://pubchem.ncbi.nlm.nih.gov/

2 http://www.rcsb.org/pdb/home/home.do

## Supplementary Material

FIGURE S1 Effects of Tan IIA, DDP, and the combination on the heart, lung, liver, kidney, and brain tissues.

## Abbreviations

2-D: two dimensional
ADM: adriamycin
CI: combination index
CID: compound ID
DDP: cisplatin
EC: esophageal cancer
ECL: electrochemiluminescence system
EMT: epithelial–mesenchymal transition
ESCC: esophageal squamous cell carcinoma
Fa: fraction affected
FCM: flow cytometry
HRP: horseradish peroxidase
NS: normal saline
PI: propidium iodide
PVDF: polyvinylidene difluoride
RMSD: root mean square deviation
tan IIA: tanshinone IIA
VEGF: vascular endothelial growth factor.
